The article "Elevated eukaryotic elongation factor 2 expression is involved in proliferation and invasion of lung squamous cell carcinoma" was retracted in 2025. Reasons: manipulated images; an official misconduct investigation; misconduct by an author; plagiarized images.

# Elevated eukaryotic elongation factor 2 expression is involved in proliferation and invasion of lung squamous cell carcinoma

**DOI:** 10.18632/oncotarget.11298

**Published:** 2016-08-16

**Authors:** Yang Song, Bing Sun, LiHong Hao, Jun Hu, Sha Du, Xin Zhou, LiYuan Zhang, Lu Liu, LinLin Gong, XinMing Chi, Qiang Liu, ShuJuan Shao

**Affiliations:** ^1^ Department of Histology and Embryology, Dalian Medical University, Dalian, China; ^2^ Department of Chest Surgery, The First Affiliated Hospital of Dalian Medical University, Dalian, China; ^3^ Institute of Cancer Stem Cell, Dalian Medical University Cancer Center, Liaoning, China; ^4^ Liaoning Key Laboratory of Proteomics, Dalian Medical University, Liaoning, China

**Keywords:** eukaryotic elongation factor 2, lung squamous cell carcinoma, proliferation, invasion, proteomics

## Abstract

Eukaryotic elongation factor 2 (EF2), is a critical enzyme solely responsible for catalyzing the translocation of the elongated peptidyl-tRNA from the A to P sites of the ribosome during the process of protein synthesis. EF2 is found to be highly expressed in a variety of malignant tumors and is correlated with cancer cell progression and recurrence. The present study was designed to uncover the function of EF2 on lung squamous cell carcinoma (LSCC) cancer cell growth and progression. Our results from clinical tissue studies showed that EF2 protein was significantly overexpressed in LSCC tissues, compared with the adjacent normal lung tissues, which was confirmed by western blotting and tissue microarray. Forced expression of EF2 resulted in the enhancement of lung squamous carcinoma NCI-H520 cells growth through promotion of G2/M progression in cell cycle, activating Akt and Cdc2/Cyclin B1. In nude mice cancer xenograft model, overexpression of EF2 significantly facilitated cell proliferation in vivo. Furthermore, forced expression of EF2 in the cells increased the capabilities of migration and invasion by changing the expressions of EMT-related proteins and genes. These results provided novel insights into the role of EF2 in tumorigenesis and progression in LSCC. EF2-targeted therapy could become a good strategy for the clinical treatment of LSCC.

## INTRODUCTION

Lung cancer is the leading cause of cancer death in the world. Lung squamous cell carcinoma (LSCC) is the second most common type of lung cancer worldwide, accounting for 30% of all lung cancers [1]. It is urgent to uncover the mechanisms underlying LSCC development. Proteomics provides a new opportunity to identify the carcinogenic mechanisms of LSCC. Fluorescent dye-labeled proteins coupled with two-dimensional gel electrophoresis (2D-DIGE) and mass spectrometric (MS) analysis have been widely applied to identify differentially expressed proteins between normal and tumor specimens [2]. These proteins could serve as early diagnosis molecular markers or prognostic indicators. In the previous research, we compared the protein profiles between LSCC tissues and adjacent normal lung tissues, and we identified a number of differentially expressed proteins by using 2D-DIGE and MS approaches [3]. Among these protein candidates, we were particularly interested in the eukaryotic elongation factor 2 (EF2), a key enzyme in the elongation step in protein translation.

Protein synthesis consists of three general steps: initiation, elongation and termination. High level protein synthesis is one of the characteristics of cancer cell metabolism [4]. The majority of translational control is exerted at the initiation stage [5], whereas specific regulation of the elongation phase also occurs under certain conditions [6–9]. However, no eukaryotic initiation factors were found in our previous study. The eukaryotic elongation factor 1 is one of eukaryotic elongation factors in eukaryote, which is involved in recruitment of aminoacyl-tRNAs onto the ribosome. It includes two subtypes, eEF1A and eEF1B. eEF1A1 and eEF1A2 are two isomers of eEF1A. eEF1B consists of one scaffold (eEF1Bγ) and two catalytic (eEF1Bα and eEF1Bβ) subunits. Their aberrant expressions are correlated with tumor cell growth, invasion, metastasis and a poor prognosis. *EEF1A2* has been recognized as an important oncogene. It is overexppressed in a number of tumors, including lung adenocarcinoma, liver cancer and pancreatic cancer [10–12]. Cancer-related overexpression of the *EEF1B2* mRNA is found in non-small cell lung cancers and esophageal carcinoma [13–14]. But we didn't identify these members of the eukaryotic elongation factor 1 in the 2D-DIGE and MS experiments.

Of particular interest is EF2, a critical enzyme that is solely responsible for catalyzing the translocation of the elongated peptidyl-tRNA from the A to P sites of the ribosome in eukaryotic tissues during translation [15]. EF2 can be inactivated via phosphorylation by EF2 kinase, which is a dedicated kinase for which EF2 is the only known substrate and binding to the ribosome is prevented, then protein synthesis is subsequently inhibited [16]. Recently EF2 is identified as a novel tumor-associated antigen [17]. It is reported that EF2 has been found to be highly expressed in a variety of malignant tumors, including human gastrointestinal cancers [18], lung adenocarcinoma [19], ovary cancer [20], hepatocellular carcinoma [21] and soft-tissue sarcomas [22]. Overexpression of EF2 is also correlated with cancer cell progression and early tumor recurrence [17–18]. These observations indicate that EF2 is probably to become an effective tumor-associated antigen target for therapy against human cancer. However, the effect of EF2 on LSCC genesis has yet not been examined and remains unknown.

The present study was designed to apply 2D-DIGE and MS approaches to identify the differential proteins in LSCC tissues with or without metastasis, using adjacent normal tissues as control. To determine the roles of EF2 in human carcinogenesis, we investigated the effects of EF2 overxpression on lung cancer NCI-H520 cell lines proliferation, morphology, cell-cycle distribution and the capability of migration. We believe these results will help to uncover the functions of EF2 in LSCC development and progression.

## RESULTS

### EF2 is highly expressed in LSCC tissues

An overlaid gel visualization image was shown in Figure 1A. Sixty-three proteins spots showed differentially expression with statistical significance (*p* < 0.05) in both metastastic and non-metastastic LSCC tissues, compared with the adjacent normal tissues. These were selected and identified following a Mascot database search using the acquired MS data. Among the differentially expressed proteins, protein spot 417 which was up-regulated (Figure 1B) by 402% and 209% (Figure 1D) in non-metastatic and metastatic LSCC tissues respectively, compared with the non-neoplastic peritumoral tissues, was identified as human EF2 (Figure 1E and Figure 1F) with a protein identification score of 65 by MS analysis. The mass signal peak was single and pillared in all of the groups (Figure 1C). The amino acid residues highlighted in bold red matched with EF2 were those detected by MS analysis (Figure 1F).

**Figure 1:** EF2 expression of LSCC tissues and peri-cacinoma lung tissues in 2-D DIGE and MS analysis **A.** Representative image of the overlaid images of Cy- labeled samples. **B.** Deep-Purple-stained gel image. The number 417 represented the protein spot of interest for EF2. **C.** The separation effect and protein content for EF2 in samples. The protein content was very high, and the separation effect was good. **D.** The expressions for protein spot EF2 in non-metastatic and metastatic LSCC tissues respectively, compared with para-carcinoma lung tissues of seven groups. SqNP, SqNT, SqMP and SqMT stand for non-metastastic para-carcinoma lung tissues, non-metastastic lung squamous cell carcinoma, metastastic para-carcinoma lung tissues and metastastic lung squamous cell carcinoma respectively. **E.** The Mascot score (65) of protein identification for spot 417 by MS. **F.** A representative tandem mass spectrum of the peptide (in red) matched for EF2 by MS.

### Western blot and IHC analysis confirm EF2 up-regulation in LSCC tissues

To confirm the proteomic result, the protein expression and distribution of EF2 in LSCC tissues were further determined by IHC and western blot analyses. We determined the EF2 protein level in a tissue microarray containing 75 paired cases of LSCC and non-neoplastic peritumoral parts. The positive degrees of immunoreactivities were measured and quantified as positive (+) or strong positive (++). Yellow, brown and brown-black grains were easily found in the cytoplasm of tumor cells in the majority of the cancer nests from LSCC patients. However, no or only small parts of yellow grains were observable in the cytoplasm of the vast majority of alveolar epithelial and bronchiolar epithelial cells in non-neoplastic peritumoral parts (Figure 2A).

**Figure 2:** EF2 expression in LSCC tissues and peri-cacinoma lung tissues by western blot and IHC analysis **A.** Representative IHC images of the EF2 protein expression in LSCC specimens and matched peri-cacinoma lung tissues of tissue microarray. P and T stand for peri-cacinoma lung tissues and LSCC tissues respectively. **B.** Western blot analysis for EF2 in 16 pairs of LSCC tissues and peri-cacinoma lung tissues. The protein level of EF2 in LSCC tissues was 4.8-fold higher than that in the peri-cacinoma lung tissues (* *p* < 0.05).

EF2 expression was only positive in 25.3% (19 of 75 cases) of non-neoplastic peritumoral parts, while it was positive in 88% (66 of 75 cases) LSCC tissues (Table 1). The average EF2 protein level in LSCC tissues was strikingly increased with statistical significance (*p*=7.5×10^-15^).

**Table 1:** EF2 expression in LSCC and peri-cacinoma lung tissues of tissue microarray

Tissues	Sum	-	+	++	Positive rate(%)	*p* value
LSCC	75	9	9	57	88	7.5×10^-15^
Peri-cacinoma lung tissues	75	56	14	5	25.3	

We further compared the protein levels of EF2 in LSCC tissues according to the classifications of tumor metastasis, pathological type, and histological grade (Table 2).

**Table 2:** Clinical characteristics and the expression for EF2 on the tissue microarray of LSCC

EF2 level	Metastasis	Non-metastasis	Pathological stages			Histological grades		
			1	2	3 and 4	Well-differentiated	moderately differentiated	poor differentiated
-	7	2	5	2	2	2	6	1
+	4	5	2	3	4	1	6	2
++	32	25	20	23	14	10	40	7
sum	43	32	27	28	20	13	52	10
Positive rate(%)	83.7	93.8	81.5	92.9	90	84.6	88.5	90.0
χ^2^	3.724		5.036			1.819		
*p*-value	0.054		0.081			0.403		

Next we performed western blotting to detect the EF2 protein expression in 16 pairs of LSCC and matched non-neoplastic peritumoral parts. Compared with matched non-neoplastic peritumoral tissues, the EF2 protein level was significantly highly expressed in tumor tissues (Figure 2B; *p*=0.0008).

### The stable overexpression of EF2 affects cell morphology

To examine the function of EF2, pcDNA3.1/myc- His(-)B-EF2 plasmid was stably transfected into NCI-H520 cells. Western blot was used to select for stable pools of cells with overexpression of the protein (the result was not shown). The cells with an empty vector were named NCI-H520/pcDB, and the two transfected cells were called NCI-H520/ pcDB-EF2-1 and NCI-H520/ pcDB-EF2-2. Compared with the control cells, NCI- H520/ pcDB-EF2 cells became larger with more elongated filopodia, as shown in Figure 3.

**Figure 3:** Cell morphology **A.** Microscopy images under the phase contrast microscope. **B.** Microscopy images by crystal violet staining. NCI-H520/pcDB-EF2 cells had larger cell shapes with more elongated filopodia than NCI-H520/pcDB cells.

### The stable overexpression of EF2 promotes the proliferation of NCl-H520 cells *in vitro*

As shown in Figure 4A, the overexpression of EF2 in NCI-H520 cells significantly promoted cell proliferation. The result was further confirmed by the colony formation assay (Figure 4B). The number of clones formed by NCI-H520/pcDB-EF2 cells remarkably increased, compared with NCI-H520/pcDB cells.

**Figure 4:** The effect of EF2 overexpression on cell proliferation of NCI- H520 *in vitro* **A.** CCK-8 assay. Transfection of EF2 significantly promoted the growth of NCI- H520/pcDB-EF2 cells. **B.** Colony formation assay. The ratio of colony formation of NCI-H520/pcDB-EF2 cells was much higher than that of NCI-H520/pcDB cells (* *p* < 0.05). **C.** FACS analysis. Cell cycle distribution was determined by the DNA content. A demonstrated decreased percentage in the G2/M phase of the NCI-H520/pcDB-EF2 cells (* *p* < 0.05). **D.** Expression of Akt1, p-Akt, p-Cylin B1, p-Cdc2, EF2 and β-actin detected by western blot.

Then we examined whether EF2 was involved in cell cycle progression. Cell cycle of the three cancer cell lines were analyzed by flow cytometry. Overexpression of EF2 significantly decreased the number of cells in the G2/M phase, while the percentages of cells in the G1 and S phase showed no significant difference between empty vector-transfected cells and EF2-transfected cells (Figure 4C). Western blot analysis showed that overexpression of EF2 increased the protein levels of phosphorylated Akt, Cdc2 and Cyclin B1 proteins (Figure 4D).

### Stable overexpression of EF2 increases migration and invasion of NCl-H520 cells *in vitro*

Cell scratch-wound assays were performed to investigate the effect of EF2 on the horizontal migration of NCI-H520 cells by observing the scratch wounding confluent monolayer of each group of cells. As shown in Figure 5A, stable overexpression of EF2 markedly increased the spreading of the NCI-H520/pcDB-EF2 cells along the edges of the wound compared with the control cells.

**Figure 5:** The effect of EF2 overexpression on cell migration and invasion **A.** Cell scratch-wound assay. At 8 h after the scratching, few cells migrated across the wound in the NCI-H520/pcDB cell groups compared with the NCI-H520/ pcDB-EF2 cell groups. At 24 h, NCI-H520/pcDB-EF2 cells reached the midline of the wound and exhibited a faster migration rate than the control group (* *p* < 0.05). **B.** Transwell migration. Significantly more NCI-H520/ pcDB-EF2 cells migrated through the basement membrane compared with NCI-H520/pcDB cells (* *p* < 0.05). **C.** Transwell invasion. Significantly more NCI-H520/pcDB-EF2 cells invaded the basement membrane compared with NCI-H520/pcDB cells (* *p* < 0.05).

Migration and invasion through a basement membrane are hallmark traits of malignancy. The modified Boyden chamber assay was performed to determine the abilities of cells to pass through the biological basement membrane. The transwell migration and invasion assays results indicated that stable overexpression of EF2 significantly promoted the capacities of migration and invasion in NCl-H520 cells *in vitro* (Figure 5B and 5C).

### Stable overexpression of EF2 has an effect on expression of EMT-related proteins and genes in NCl-H520 cells *in vitro*

The protein levels of E-cadherin, β-catenin, Vimentin and MMP2 were examined by western blot. Overexpression of EF2 resulted in a reduction of E-cadherin and a raise of Vimentin and MMP2. The levels of β-catenin protein were similar among the three cell lines (Figure 6A). Furthermore, we analyzed the expression of genes related to EMT including *SNAIL*, *TWIST* and *FOXC1* by qPCR. The results showed that overexpression of *EF2* promoted the expressions of *SNAIL* and *TWIST*, while it inhibited the expression of *FOXC1* (Figure 6B).

**Figure 6:** The effect of EF2 overexpression on the expressions of EMT-related proteins and genes in NCl-H520 cells **A.** The expression of β-catenin, E-cadherin, MMP2, Vimentin, EF2 and β-actin by western blot. **B.** The expressions of *SNAIL*, *TWIST* and *FOXC1* detected by qPCR in three groups of the cells (* *p*<0.05). **C.** Representative IHC images of E-cadherin, Vimentin and MMP2 in EF2 positive clinical 22 pairs of LSCC and non-neoplastic peritumoral parts.

To confirm the result that EF2 overexpression affected expression of EMT-related protein, E-cadherin and other EMT markers were analyzed in 22 pairs of EF2 positive LSCC and their matched non-neoplastic peritumoral parts by IHC staining. Vimentin and MMP2 proteins were detected in 81.8% (18 of 22) and 72.7% (16 of 22) of LSCC, while they were positive in 31.8% (7 of 22) and 27. 3% (6 of 22) of non-neoplastic peritumoral parts respectively. Yellow, brown and brown-black grains were easily observed in the cytoplasm of the cancer cells at the cancer nests of LSCC tissues. However no yellow or only buffy grains were found in most of the alveolar epithelial cells in their paired adjacent normal lung tissues. The positive rate of E-cadherin protein was 27.3% (6 of 22) in LSCC and 86.4% (19 of 22) non-neoplastic peritumoral parts. Buffy, brown and brown-black grains were detected in the alveolar epithelial cells in their paired adjacent normal lung tissues. Whereas cytoplasm of the tumor cells was negatively or weakly positive stained in the majority of the cancer nests (Figure 6C). Vimentin and MMP2 protein levels in LSCC were increased, and E-cadherin protein level was decreased in tumor tissues.

### Overexpression of EF2 enhances tumorigenicity of NCI-H520 cells *in vivo*

To examine whether overexpression of EF2 promoted tumorigenicity *in vivo*, EF2/pcDNB3.1 and pcDNB3.1 vector-transduced NCI-H520 cells were subcutaneously injected into the left flank of each nude mice and tumor volume was examined daily. Twelve weeks later, we observed that the NCI-H520/pcDB cells only growed into very small tumors compared with that of NCI-H520/pcDB-EF2 cells (Figure 7).

**Figure 7:** Overexpression of EF2 enhances the tumorigenicity of NCI-H520 cells In nude mice, the NCI-H520/pcDB-EF2 cells grew larger tumors compared with the control group.

## DISCUSSION

In the present study, we used the proteomic approach to investigate the differentially expressed proteins between LSCC tissues and adjacent normal tissues. EF2 was identified as the differential protein and highly expressed in LSCC. The result was confirmed by western blotting and tissue microarray.

EF2 is the critical enzyme governing the elongation of nascent proteins which is responsible for the translocation of ribosome along the specific mRNA during translation. Overexpression of EF2 is observed in various cancers, including lung adenocarcinoma [17–18]. It was reported that EF2 was highly expressed in lung adenocarcinoma and it was positively correlated with a significantly higher incidence of tumor recurrence and increased cisplatin resistance, which ultimately reflected in a worse prognosis [19]. The research also showed that small ubiquitin-related modifier (SUMO)-1 activating enzyme subunit 2(SAE2) might play an important role during this process. Posttranslational modifications (PTMs) of proteins are involved in multiple biological processes, such as gene regulation, cellular function, tissue development, and metabolism, whose alterations trigger occurrence of cancers and other diseases. PTMs includes enzymatic changes such as ubiquitin (Ub), SUMO, phosphor, acetyl and methyl moieties [23–24]. SAE2 is one of enzymes for sumoylation in which SUMO protein moiety is enzymatically conjugated to a substrate protein [25–26]. SAE2 was highly expressed in lung adenocarcinoma tissues and cell lines which might be concomitantly expressed with EF2 to increase the efficacy of sumoylation and to maintain EF2 stability.

A wide range of alterations in gene expression have been identified in lung cancers, but the mechanisms of EF2 upregulation in LSCC are not clear. It is believed that proliferating cells, such as cancer cells, increase protein synthesis to support growth-related anabolic processes [27]. Akt is a serine/threonine kinase which mediates a variety of biological processes. And activation of Akt is considered to play an important role in tumorigenesis. Akt pathway is vital to growth-factor stimulation of mammalian target of rapamycin (mTOR) signaling through inactivation of TSC2, an upstream regulator of mTOR [28], resulting in activation of EF2 through the inactivation of the EF2 kinase. Our results demonstrated that elevated expression of EF2 in LSCC activated Akt. We believed that Akt might be a significant molecule in LSCC tumorigenesis which promoted cancer cell growth. Cdc2/Cylin B1 are important G2/M regulators. Overexpression of EF2 in LSCC significantly promoted cell growth *in vitro* and *in vivo* through the acceleration of the G2/M progression in the cell cycle, through activation of Cdc2/Cylin B1. Our findings supported the observations of Nakamura [18], indicating that elevated expression of EF2 could facilitate LSCC cell growth.

We also found that overexpression of EF2 in NCI-H520 cells enhanced the capabilities of migration and invasion, suggesting that EF2 was probably involved in tumor metastasis. It was reported that highly expression of EF2 was significantly correlated with node positivity of receptor-positive breast cancer [29]. Sun HG [30] showed that the levels of EF2 in the serum of NSCLC patients were markedly higher in stages III and IV than stages I and II. Metastasis is a very complex biological process in carcinomas. The mechanisms of this process still remain largely unknown. Recently, many researches show that activation of the ‘epithelial-mesenchymal transition’ (EMT) is detrimental to the dissemination and invasion of certain cancer cells [31]. During EMT, epithelial tumor cells lose their epithelial traits, such as E-cadherin and β-catenin, instead they display fibroblast-type traits such as Vimentin [32–33]. MMP2 is one membrane of matrix metalloproteinases (MMPs), which is capable of degrading type IV collagen and some bioactive molecules of the extracellular matrix and helps increase the invasive potential of tumor cells. In the present study overexpression of EF2 inhibited the expression of E-cadherin and increased the levels of Vimentin and MMP2 proteins in NCI-H520/pcDB-EF2 cells. We also examined the mRNA levels of *SNAIL*, *TWIST* and *FOXC1*, transcription factors involved in EMT [34–38]. The qPCR results were consistent with their elevated migration and invasion capabilities *in vitro*. Moreover, morphological studies confirmed the results above. The cells became larger with more filopodia after stably transfected with *EF2*, which suggested that overexpression of EF2 might cause morphological transformation from epithelial cells to mesenchymal cells. Taken together, we hypothesized that EF2 may promote the development of LSCC metastasis by changing the expressions of EMT-related proteins and genes. But further investigations are needed to confirm whether EF2 is a decisive gene for promoting EMT in tumor cells.

In conclusion, we found that EF2 was highly expressed in LSCC, which may be the results of the characteristics of cancer cell metabolism in cancer cells. Further more, elevated expression of EF2 could facilitate LSCC cell growth, migration and invasion. These results provide novel insights into the role of EF2 in tumorigenesis and progression in LSCC. EF2 has certain clinical values for early diagnosis of LSCC and could be used as a tumor-associated antigen in cancer research. EF2-targeted therapy is probably to become a good therapeutic strategy and inhibition of protein synthesis may be an underlying mechanism for the clinical treatment of LSCC.

## MATERIALS AND METHODS

### Ethics statement

All the tissue samples and patient data used in the study were obtained from the First and Second Affiliated Hospital of Dalian Medical University. The patients understood the collecting process, purpose of the specimen, and signed informed consent for specimen collection. All the data used in this study was anonymized. Mice were obtained from Dalian Medical University Laboratory Animal Center. We anesthetized the mice by CO_2_ and then froze them at 4°C. All the animal and human experiments were approved by the Medical Ethics Committee of Dalian Medical University.

### Specimen collection and proteomic analysis

The tissue samples and patient data used in the study were obtained during surgery from LSCC patients (six male and one female) with an age range of 36 to 67 years, at the Department of Chest Surgery at the First and Second Affiliated Hospital of Dalian Medical University from March 2004 to December 2006. Among the specimens, three pairs were non-metastastic and four pairs were metastatic. Two cases were poorly differentiated disease, three cases were moderately differentiated disease, and two cases were well-differentiated LSCC. None of the patients received preoperative radiotherapy or chemotherapy. Neoplastic and non-neoplastic peritumoral samples (> 5 cm away from the lesion) were immediately frozen and stored at −80°C. Pathological diagnoses were performed on all specimens to confirm that the tumor specimens were real LSCC tissues. Surgery follow-ups were conducted with each patient annually for three years.

To prepare protein extracts, the tissues were homogenized in a buffer containing 30 mM Tris, 2 M thiourea, 7 M urea, 4% CHAPS and a cocktail of protease inhibitors (GE Healthcare, USA) and sonicated on ice. The supernatants were collected by centrifugation at 12,000 g for 15 min at 4°C. For 2D-DIGE, 50 μg of pooled protein was labeled with Cy2 as the internal standard control; Cy3 and Cy5 were used to label experimental samples. The samples were separated bi-dimensionally with 12.5% SDS-PAGE gels. Images were acquired by using the fluorescence scanner (GE Healthcare, USA) through excitation wavelengths of 488/520 nm, 532/580 nm or 633/670 nm, respectively. Gel image analysis was processed using DeCyder 6.5 software (GE Healthcare, USA). The BVA software module was used for gel-to-gel and average abundance spot and statistics calculations. The protein abundance was represented by the volume ratio of the samples versus the standards (based on the standard normalization). The spots for proteins of interest with an average ratio greater than 1.50 or less than −1.50 (*p* <0.05) at the 95% confidence level were selected for protein identification by mass spectrometer (Bruker Daltonics, Germany). The resulting peptide and the corresponding fragmentation spectra were searched against the Homo sapiens database derived from the NCBInr database, then analyzed using the MASCOT search engine (Matrix Science, UK).

### Western blotting and LSCC tissue microarrays analysis

Approximately 50 μg of protein from each of the 16 pairs of LSCC tissues with the non-neoplastic peritumoral parts were resolved in 8% SDS-PAGE (Bio-Rad, USA) After gel electrophoresis and membrane transfer, the membrane was probed with rabbit anti-EF2 monoclonal antibody (1:1000, EPITOMICS, China) and mouse anti-actin monoclonal antibody (1:3000, Proteintech Group, China). The secondary antibodies used were goat anti-rabbit or goat anti-mouse IgG conjugated to horseradish peroxidase (1:2000, Golden Bridge, China).

The LSCC microarrays were purchased from Chaoxin Biotechnology Co., China. The arrays contained 75 paired cases of LSCC and separate, matched adjacent lung tissues. Strict pathological diagnoses and post-operative follow-ups were performed for all patients. Immunohistochemical analysis was performed according to the following procedures. Briefly, the tissue arrays were deparaffinized, rehydrated and microwaved. Then, the tissue arrays were incubated with rabbit anti-EF2 monoclonal antibody (1:50) overnight at 4°C, followed by a biotinylated secondary antibody and peroxidase-labeled streptavidin complex detection (Golden Bridge, China). The localization and distribution of the EF2 were visualized by examining the slides under a microscope (Nikon, Japan).

Positive immunoreactivity was observed in the cell cytoplasm in the majority of LSCC cancer nests. The positive degree of the immunoreactivity was determined by the score of the grade defined by the percentage of positive cells in the total cancer cells or in the bronchiolar and alveolar epithelial cells, as well as by the score of the staining intensity of positive cells. The scores (score I) of 0, 1, 2, 3 and 4 were granted by the percentages of positive cells which ranged from 0 to 5% (grade 0), 5% to 25% (grade 1), 25% to 50% (grade 2), 50% to 75% (grade 3), and 75% to 100% (grade 4). The staining intensities of positive cells were scored as 0, 1, 2 and 3 (score II) for the positive signals that appeared as negative, the pallide-flavens grains, the buffy grains and the brown-black grains in the cell cytoplasm. Finally, the product (score III) of scores I and scores II was used to define the EF2 expression intensity in the tissues. The values of score III ranged from 0 to 4, 5 to 8 and 9 to 12 and represented a negative, moderate and high expression of EF2 in the corresponding tissues, respectively.

### Cell culture and stable overexpression of EF2 in NCI-H520 cells

The human lung squamous carcinoma NCI-H520 cells (ATCC® HTB182^TM^) were pursued from Cancer Hospital Chinese Academy of Medical Sciences and cultured with RPMI 1640 media (Invitrogen, USA) supplemented with 10% fetal bovine serum at 37°C with 5% CO_2_. Cells were passed in culture no more than 2 months. The expression vector for *EF2* was constructed by inserting CDS sequence (2577bp, Nucleotide of *EF2*: BC126259) into the XhoI/ HindIII sites in pcDNA3.1/myc-His(-)B vector (Vigorous Biotechnology Beijing Co., Ltd.). The primer sequences of *EF2* were as follows: forward primer: 5′- ccgCTCGAGcaccATGGTGAACTTCACGGTAGACCAG-3′, reverse primer: 5′- cccAAGCTTCTACAATTTGTCCAGGAAGTTGTCC-3′. pcDNA3.1/myc-His(-)B and pcDNA3.1/myc-His(-)B-EF2 plasmids were transfected with Lipofectamine 2000 (Invitrogen, USA) into the NCI-H520 cell lines according to the kit instructions. The transfected cells were selected with 400 μg/mL G418 (Invitrogen, USA). After approximately eight weeks of selection, the cells were harvested for use and cryopreserved. The stable transfected cells with overexpression of EF2 were confirmed by qPCR and western blot analysis and used for further research.

### Cell morphology analysis

The cells were cultured in six-well plates. After fixation in ice-cold 70% methanol for 10 min, 0.1% crystal violet was added into the culture for 5 min. The cells were washed with PBS, and then, cell morphology was examined under microscope. Meanwhile, cell morphology was also captured under the phase contrast microscope with a digital camera (Nikon, Japan).

### Growth curves, colony formation assays and cell cycle analysis by flow cytometry

Growth curves were performed using a CCK-8 assay kit (Dojindo Laboratories, Tokyo, Japan) according to the manufacturer's instructions. Briefly, 5×10^3^ cells were seeded in 96-well plates in RPMI-1640 medium. The culture medium was removed and 100 μL of fresh culture medium containing 10 μL of CCK-8 were added to each well. The cells were then incubated at 37°C for 1 h. At 0, 24, 48, 72 and 96 h, the optical density values were measured against a reagent blank at a test wavelength of 450 nm. A total of 4×10^2^ cells were plated in 100 mm culture dishes. After 14 day incubation, the cells were fixed with 70% methanol and stained with 0.1% crystal violet, and colonies of > 50 cells were manually counted. All experiments were performed in independent triplicate.

Cells were cultured with 2×10^5^ cells in each six-well plate as described above and harvested after 24 h. Cells were trypsinized, washed with PBS twice and then fixed with cold 70% ethanol at 4°C overnight. For flow cytometric analysis, the cells were treated with RNase A for 30 min at 37°C, stained with propidium iodide (PI) solution for 30 min at 4°C and then measured by flow cytometry (BD FACS Caton, USA). ModFit LT software was used for data acquisition and analysis.

### Wound healing, migration and invasion assays

The cells were seeded in six-well plates using 10% fetal bovine serum until confluence. A wound area was generated by scraping with a 200 μl pipette tip. Then, the cells were cultured in serum-free medium. After 8 h and 24 h, cells in the wounded monolayer were counted randomly at multiple fields. The fields were photographed using a phase contrast microscope.

Cell invasion and migration were assessed using transwell chambers (Costar, USA). 5×10^5^ cells were resuspended with 0.5 mL of serum-free medium and added to the wells of an 8 μm pore polycarbonate membrane, either coated with (for invasion assays) or without (for migration assays) 3 μg/μl Matrigel (Sigma, USA). The lower chambers were filled with 200 μl of RPMI1640 containing 0.1 μg/μl of fetal bovine serum. The plates were incubated at 37°C for 18 h for migration and 24 h for invasion. The number of cells with 0.1% crystal violet staining on the undersurface of the polycarbonate membranes was counted at least 6 unbiased (200×) fields. The assays were performed in triplicate and the mean cell numbers and standard deviations were calculated.

### RNA extraction and quantitative real-time reversed transcription-PCR

Total RNA was exacted using the Aqua Pure RNA Isolation reagent (Invitrogen, USA) according to the manufacturer's instructions. Then, it was reverse transcribed to cDNA by using of a transcript cDNA synthesis Kit (Agilent, USA). The cDNA (500 ng), mixed with SYBR green PCR master mix (Agilent, USA), was used for real-time quantitative-PCR with stratagene Mx3000P (Agilent, USA). The primer sequences were *SNAIL*, forward 5′-ATCGGAAGCCTAACTACAGC-3′, and reverse 5′-CAGAGTCCCAGATGAGCATT-3′; *TWIST*, forward 5′-GGAGTCCGCAGTCTTACGAG-3′, and reverse 5′-TCTGGAGGACCTGGTAGAGG-3′; *FOXC1*, forward 5′-TAAGCCCATGAATCAGCCG-3′, and reverse 5′-GCCGCACAGTCCCATCTCT-3′; *EF2*, forward 5′-CTGCCGAGCGGGCCAAGAAA-3′, and reverse 5′-CGGGGCTGGTGGCTGACTTG-3′; and *β-actin*, forward 5′-CCTCTCCCAAGTCCA CACAG-3′ and reverse 5′-GGGCACGAAGGCTCATCATT-3′.

### Western blotting analysis

Protein extraction and western blotting were performed as described previously. β-actin was used as the internal standard control. The membranes were probed with antibodies to Akt1(10176-2-AP, ProteinTech Group; 1: 400), E-cadherin (20874-1-AP, ProteinTech Group; 1:800), β-catenin(17565-1-AP, ProteinTech Group; 1:3000), MMP2(BS1236, BioWorld Technology, Inc., USA; 1:200), p-Akt(S473)(BS4007, BioWorld Technology, Inc., USA; 1:200), p-Akt(T308)(AP0056, BioWorld Technology, Inc., USA; 1: 200), p-Cyclin B1(S126)(BS4225, BioWorld Technology, Inc., USA; 1:400), p-Cdc2(T161) (BS4033, BioWorld Technology, Inc., USA; 1:400) and Vimentin (V6389, Sigma, USA; 1:1000).

### Immunohistochemistry(IHC) analysis of EMT-related proteins

The expressions of E-cadherin and other EMT markers in EF2 positive clinical 22 pairs of LSCC and non-neoplastic peritumoral parts were analyzed by IHC staining. IHC staining was performed as previously described in the LSCC tissue microarrays analysis procedures. The tissues were incubated with E-cadherin (1:300), MMP2(1:200)and Vimentin (1:50) overnight at 4°C. The positive reaction was manifested as a brown stain. The randomly selected sections were scanned at 100× and 400× magnification to visualize the localization and density of the positive reaction.

### Xenografting nude mice

To examine the *in vivo* tumorigenicity of NCI-H520 cells with overexpression of EF2, six-week-old male nude mice were purchased and allowed to acclimate one week in the animal facility. 10^7^ cells were subcutaneously injected into the left flank of nude mice. The mice were checked daily for tumor growth, anesthetized and sacrificed by CO_2_ after 12 weeks. The xenografted tumors were examined.

### Statistics

All statistical analyses were performed using SPSS 13.0 software. Data were presented as the mean ± standard deviation (S.D.). The associations between EF2 expression and clinicopathologic features of LSCC were analyzed using chi-square tests and Fisher's exact test. The one-way analysis of variance (ANOVA) test and Student Newman Keuls method were used between the two comparisons among all groups. Statistical significance was set at *p* < 0.05.
